# Sirtuin1 single nucleotide polymorphism (A2191G) is a diagnostic marker for vibration-induced white finger disease

**DOI:** 10.1186/1868-7083-4-18

**Published:** 2012-10-01

**Authors:** Susanne Voelter-Mahlknecht, Bernd Rossbach, Christina Schleithoff, Christian L Dransfeld, Stephan Letzel, Ulrich Mahlknecht

**Affiliations:** 1 Institute of Occupational, Social and Environmental Health, University of Mainz, Obere Zahlbacher Strasse 67, D-55131 Mainz, Germany; 2 Institute of Occupational Medicine, Social Medicine and Health Services Research, University of Tuebingen, Wilhelmstrasse 27, D-72074, Tuebingen, Germany; 3 Department of Internal Medicine, Division of Immunotherapy and Gene Therapy, José Carreras Research Center Saarland, University Medical Center, D-66421, Homburg/Saar, Germany

**Keywords:** Epigenetics, Hand-arm vibration syndrome (HAVS), Sirtuins, Vibration-induced white finger disease (VWF)

## Abstract

**Background:**

Vibration-induced white finger disease (VWF), also known as hand-arm vibration syndrome, is a secondary form of Raynaud’s disease, affecting the blood vessels and nerves. So far, little is known about the pathogenesisof the disease. VWF is associated with an episodic reduction in peripheral blood flow. Sirtuin 1, a class III histone deacetylase, has been described to regulate the endothelium dependent vasodilation by targeting endothelial nitric oxide synthase. We assessed Sirt1single nucleotide polymorphisms in patients with VWF to further elucidate the role of sirtuin 1 in the pathogenesis of VWF.

**Methods:**

Peripheral blood samples were obtained from 74 patients with VWF (male 93.2%, female 6.8%, median age 53 years) and from 317 healthy volunteers (gender equally distributed, below 30 years of age). Genomic DNA was extracted from peripheral blood mononuclear cells and screened for potential Sirt1single nucleotide polymorphisms. Four putative genetic polymorphisms out of 113 within the Sirt1 genomic region (NCBI Gene Reference: NM_012238.3) were assessed. Allelic discrimination was performed by TaqMan-polymerasechainreaction-based allele-specific genotyping single nucleotide polymorphism assays.

**Results:**

Sirt1single nucleotide polymorphism A2191G (Assay C_25611590_10, rs35224060) was identified within Sirt1 exon 9 (amino acid position 731, Ile → Val), with differing allelic frequencies in the VWF population (A/A: 70.5%, A/G: 29.5%, G/G: 0%) and the control population (A/A: 99.7%, A/G: 0.3%, G/G: 0.5%), with significance levels of *P* < 0.001 (Mann–Whitney *U* test (two-tailed) *P* <0.001; F-exact *t*-test and Chi-square test with Yates correction (all two-tailed): *P* <0.0001). The heterogeneous A/G genotype in base pair position 2191 is significantly overrepresented in the VWF patient population when compared with healthy controls.

**Conclusion:**

We identified theSirt1_A2191G_single nucleotide polymorphism as a diagnostic marker for VWF.

## Background

Vibration-induced white finger disease (VWF) is an industrial injury that is triggered by the continued use of vibrating hand-held machinery. The disease is a widespread and officially recognized occupational disease affecting tens of thousands of employees. According to data that have been published by the Medical Research Council, around 2 million people in Britain are continuously subjected to potentially harmful levels of hand-arm vibration and around 300,000 people are anticipated to suffer from moderate to severe finger blanching (VWF) linked to such exposure, which may lead to considerable time off work, early retirement and considerable payouts from civil compensation schemes. In fact, a UK government fund that had been set up to cover claims by ex-coalminers who were exposed to the use of vibrating hand-held machinery had exceeded £100 million in payments by 2004 [1].

VWF is characterized by vasospastic attacks and a cold sensation in the fingers followed by cyanotic discoloration or skin pallor (Figure 1) [2-5]. In addition, the sensitivity in the affected fingers is usually reduced. As a consequence, some of the affected individuals have difficulty carrying out manual activities because of their limited fine motor skills. Attacks may be associated with a tingling sensation, feeling loss, stiffness and at times even severe pain. In an early stage of the disease, vasospastic attacks occur particularly under the influence of low temperature. In later stages of the disease, a cold ambient temperature is no longer required as a trigger to cause vasospasm. VWFmay be triggered by hand-operated technical tools and machines that cause high frequency vibration with an oscillation rate >50 Hz. The occurrence of the disease depends on the length and intensity of daily exposure to vibration. To date, little is known about individual susceptibility factors with respect to VWF. 

**Figure 1:** Hands of a person suffering from vibration-induced white finger disease.

The pathogenesis of this disease is currently unclear. Epigenetics is gaining increasing importance in the understanding of numerous diseases. Epigenetic pathways have recently been suggested to be important in the regulation of vascular gene expression in the pathophysiology of atherosclerosis [6,7], the microvascular environment of tumors [8], cytokine-inducible gene expression in vascular endothelium [9], and in the developmental regulation of vascular remodeling [10,11]. Chromatin-based regulatory mechanisms may therefore play a key role in the constitutive expression of endothelium-restricted genes [10].

A single nucleotide polymorphism (SNP) is defined as the difference between chromosomes in the base present at a particular site in the DNA sequence that naturally occurs within a population, and presents the most common type (90%) of genetic variation in humans [12]. Hopefully, increasing knowledge of an individual’s SNP genotype may contribute to the assessment of disease susceptibility and individualized treatment modalities [13].

Based on structural and functional similarities, mammalian histone deacetylases (HDACs) are grouped into four categories. There are three classes of non-sirtuin HDACs, comprising the yeast HDACright parietal dorsal 3 homologs (class I HDACs); class II HDACs, which share a significant degree of homology with the yeast HDA1; and the most recently described class IV HDACs, which comprise HDAC11-related enzymes. There is one class of sirtuin HDACs (class III HDACs), which are homologs to the yeast Sir2 protein.

The yeast Sir2 protein has seven human homologs (SIRT1-7), which play a central role in epigenetic gene silencing, DNA repair and recombination, cell-cycle, microtubule organization, and in the regulation of aging [14].

SIRT1, which is a member of the Sir2 family of NAD^+^-dependent HDACs, deacetylates histone H3 lysines 9 and 14 and specifically histone H4 lysine-16, while it hydrolyzes one molecule of NAD^+^ for every lysine residue that is deacetylated [14,15]. Derivatives of the yeast Sir2 HDAC share a common catalytic domain, which is highly conserved in organisms ranging from bacteria to humans and which is composed of two distinct motifs that bind NAD^+^ and the acetyl-lysine substrate, respectively [14-17]. SIRT1 is known to directly modify chromatin and to silence transcription, to modulate the meiotic checkpoint, and as a probable antiaging effect, to increase genomic stability and to suppress recombinant DNA recombination [18,19]. While, for yeast Sir2, no targets are known apart from histones, SIRT1 has a large and still growing list of targets,including p53 and forkhead transcription factors, which are mammalian homologs of Daf-16 and which are known to function as sensors of the insulin signaling pathway [14,18].

## Results and discussion

Within the Sirt1 genomic sequence, 113 potential SNPs were identified, of which six were coding nonsynonymous SNPs. Three out of six were found to be false-positive SNPs, but four out of six were further analyzed in patients with VWF in relation to healthy controls. While rs1063114 and rs1063112 were in fact identified to be false positive SNPs, we confirmed rs1063111, rs35224060, rs3740051 and rs2236319 to be true SNPs. For rs1063111, we had identified a frequency of 99.5% for the T/T allele and 0.5% for the A/T allele in the control population, which remained unchanged in the VWF patient population. Because the T/T allele had a frequency of 98.3% versus 1.7% for the A/T allele in the HapMap data for Central Europeans, this SNP may be considered a true SNP, which remains unchanged within the VWF population. Important details regarding rs3740051, the Sirt1 promoter SNP located 521 bp upstream of the translational start codon, also need to be mentioned.In the Central European Caucasian population, we identified a 90% frequency for the A/A genotype, 9.5% for the A/G genotype and an allelic frequency of 0.5% for the G/G genotype. This is in accordance with the HapMap data and showed no difference in the population of patients with VWF. However, the HapMap allelic reported for the Indian (A/A: 98.0%, A/G: 1.0%, G/G: 1.0%), Chinese (A/A: 51.1%, A/G: 35.6%, G/G: 13.3%) and Japanese (A/A: 38.6%, A/G: 56.8%, G/G: 4.5%) populations is remarkable divergent, a fact that is currently unexplained. Similar observations have been made for the Sirt1 intron 4 SNP rs2236319: Central European Caucasian population -A/A: 90.0%, A/G: 8.3%, G/G: 1.7%, with no difference between the control population and the VWF population; Chinese population- A/A: 51.1%, A/G: 35.6%, G/G: 13.3%, which is identical to the rs3740051 distribution; and Japanese population - A/A: 31.8%, A/G: 63.6%, G/G: 4.5%, which is also noteworthy and currently without explanation. The most striking results have however been obtained for rs35224060, the Sirt1 SNP A2191G (Assay C_25611590_10) that was identified within Sirt1 exon 9 (amino acid position 731, Ile → Val), with differing allelic frequencies in the VWF population (A/A: 70.5%, A/G: 29.5%, G/G: 0%) and the control population (A/A: 99.7%, A/G: 0.3%, G/G: 0.5%) with significance levels of *P* < 0.001 (Mann–Whitney *U* test (two-tailed) *P* < 0.001; F-exact *t*-test and Chi-square test with Yates correction (all two-tailed): *P* < 0.0001 respectively). The heterogeneous A/G genotype in bp position 2191 is significantly overrepresented in the VWF patient population when compared with healthy controls (Table 1).

**Table 1:** Comparison of the allelic distribution of patients with vibration-induced white finger disease and healthy controls

**dbSNP [Assay ID]**	**Patients with VWF**			**Healthy controls**		
**rs1063114**	Allele A/A: 0/74	Allele A/T: 0/74	Allele T/T: 74/74	Allele A/A: 0/203	Allele A/T: 0/203	Allele T/T: 203/203
[C_9638456_10]	(0%)	(0%)	(100%)	(0%)	(0%)	(100%)
**rs1063111**	Allele A/A: 0/74	Allele A/T: 0/74	Allele T/T: 74/74	Allele A/A: 0/200	Allele A/T: 1/200	Allele T/T: 199/200
[C_9638445_10]	(0%)	(0%)	(100%)	(0%)	(0.5%)	(99.5%)
**rs1063112**	Allele C/C: 0/49	Allele C/T: 0/49	Allele T/T: 49/49	Allele C/C: 0/299	Allele C/T: 0/299	Allele T/T: 299/299
[SIRT1-A485]	(0%)	(0%)	(100%)	(100%)	(0%)	(100%)
**rs35224060**	Allele A/A: 52/74	Allele A/G: 22/74	Allele G/G: 0/74	Allele A/A: 316/317	Allele A/G: 1/317	Allele G/G: 0/317
[C_25611590_10]	(70.5%)	(29.5%)	(0%)	(99.7%)	(0.3%)	(0%)
**rs3740051**						
[C_27471644_10]	Allele A/A: 62/68	Allele A/G: 6/68	Allele G/G: 0/68	Allele A/A: 170/189	Allele A/G: 18/189	Allele G/G: 1/189
**Sirt1 promoter**	(91%)	(9%)	(0%)	(90%)	(9,5%)	(0.5%)
**rs2236319**						
[C_15954063_10]	Allele A/A: 58/66	Allele A/G: 8/66	Allele G/G: 0/66	Allele A/A: 171/193	Allele A/G: 22/193	Allele G/G: 0/193
**Sirt1 Intron 4**	(88%)	(12%)	(0%)	(88%)	(12%)	(0%)

dbSNP: Database of Single Nucleotide Polymorphisms; VWF: vibration white finger disease.

To date, little is known about the pathogenesis of VWF. It is however widely accepted that both the nervous and the vascular systems are affected and that vasoconstrictive effects dominate over vasodilatative effects during a vasospastic attack. In this process, endothelium-dependent and endothelium-independent mechanisms regulating the vascular tone may be distinguished. The endothelium-dependent vascular regulation is based on the interplay of competing vasoconstrictive and vasodilatative substrates, of which nitric oxide (NO), a factor that significantly depends on the activity of the endothelial isoform of NO synthase (eNOS, synonym: NOS3), is a key player.

There is increasing evidence that epigenetic mechanisms play a key role in a number of vascular disorders [10,20]. SIRT1 and eNOS co-localize and co-precipitate in endothelial cells, and SIRT1 deacetylates eNOS, thus stimulating eNOS activity, which subsequently increases endothelial NO [21]. Fully functional Sirt1 is essential in the regulation of endothelium-dependent vasodilation and may have profound effects not only on the control of the local vascular tone and systemic blood pressure, but also in the pathogenesis of VWF.

## Conclusions

Our study shows an important, highly significant accumulation of the heterogeneous genotype of the Sirt1 SNP A2191G (Ile → Val) when compared with healthy controls (*P* <0.001).

We therefore claim the Sirt1_2191_ A/G genotype to be a risk factor for VWF, and that it may be used as a biological marker to facilitate the identification of risk populations who are being considered for exposure to potentially hazardous hand-held vibrating machinery. This may prevent thousands of employees from experiencing physical pain and disability, in addition to long-lasting administrative fights for VWF compensation, which frequently end unsettled and in great frustration.

## Methods

### Patients and control group

Peripheral blood samples were obtained from 74 patients with VWF and from 317 healthy volunteers. Informed consent was given and the study was approved by the local ethics committee. The patient group was composed of 69 male (93.2%) and five female (6.8%) patients with a median age of 53 years, ranging from 29 to 74 years; the gender contribution is caused by a higher frequency on VWF in men and reflects the real world gender distribution of the disease. In the control group, genders were equally distributed (all below the age of 30 years). Genomic DNA was extracted from 5 mL peripheral EDTA (ethylenediaminetetraacetic acid)-blood with the FlexiGene DNA Kit (Qiagen, Hilden, Germany) according to the manufacturer’s instructions. DNA quantification was carried out on a Nanodrop ND-1000 Spectrophotometer (Peqlab Biotechnologie GmbH, Erlangen, Germany). Samples were then stored in double diluted H_2_O at −20°C.

### *In silico* analysis

Based on *in silico* expression analyses with the EST profile viewer (National Center for Biotechnology Information (NCBI)), a strong overexpression of Sirt1 was observed in vascular endothelial cells. In addition, we had observed increased Sirt1 expression levels in response to the NO liberator sodium nitroprusside in earlier analyses [22]. Since VWF results from episodic reduction in peripheral blood flow in response to occupational exposure to hand-held vibrating machinery, and Sirt1 has been reported to promote endothelium-dependent vasodilation by targeting eNOS [21], we screened the Database of Single Nucleotide Polymorphisms (dbSNP; NCBI) [23], the HapMap database [24] and the Applied Biosystems database (TaqMan SNP Genotyping Assays, Applied Biosystems, Life Technologies Corporation, 5791 Van Allen Way, PO Box 6482 Carlsbad, California 92008 [25] for potential Sirt1 SNPs in order to further elucidate the role of Sirt1 in the pathogenesis of VWF. We focused our search criteria on coding nonsynonymous SNPs, in addition to a Sirt1 intron 4 SNP and a Sirt1 promoter SNP. As the HapMap data are publicly released to dbSNP, we performed our search mainly via dbSNP and the Applied Biosystems database, which both included HapMap data.

### Genotyping

Four putative genetic polymorphisms out of 113 within the Sirt1 genomic region (NCBI Gene Reference: NM_012238.3) were assessed on genomic DNA from patients with VWF and from healthy volunteers by real-time PCR. Allelic discrimination was performed by TaqMan-PCR-based allele-specific genotyping SNP-assays C_9638456_10 (NCBI SNP reference: rs1063114, exon 8), C_9638445_10 (NCBI SNP reference: rs1063111, exon 8), SIRT1-A485 (NCBI SNP reference: rs1063112, exon 8), C_25611590_10 (NCBI SNP reference: rs35224060, exon 9), C_27471644_10 (NCBI SNP reference: rs3740051, Sirt1 promoter) and C_15954063_10 (NCBI SNP reference: rs2236319, intron 4) as provided by the manufacturer (Applied Biosystems) (Table 2). PCR reactions and allele detection were done in duplicate and carried out in 96-well plates on an ABI PRISM 7000 Thermocycler (Applied Biosystems) and the ABI PRISM 7000 SDS software was used. For one PCR reaction (5 μL/well), 2.5 μL TaqMan PCR Amplification Mix (2× TaqMan PCR Amplification Mix, No AmpErase UNG, Applied Biosystems) and 0.25 μL of the 20× SNP Genotyping Assay Mix (4 μM probe, 18 μM primer, Applied Biosystems) were added to each well and 2.25 μL DNA (5 ng) were added. Every single run (96-well plate) included two no-template controls, a positive control (for Sirt1, *BAC genomic clone RZPDB737C042021D*) and 317 different DNA samples from healthy volunteers. After preincubation of the reaction mixture at 95°C for 10 min, thermocycling was carried out at 92°C for 15 s and 60°C for 1 min for a total of 60 cycles. To discriminate allelic differences, fluorescence intensities of the reporter dyes VIC and FAM were read relative to the fluorescence intensity of a passive reference dye (ROX), which then yielded specific normalized reportervalues. In order to correct fluctuations in the optical quality of the reaction tubes that have been used, signal intensities that were measured prior to PCR were subtracted from the values that were measured after PCR (postread – preread).

**Table 2:** Overview of the potential nonsynonymous Sirt1 SNPsin silico and analyzed

**dbSNP [Assay ID]**	**Region**	**5 **^**′ **^**Near Seq 30 bp**	**Allele**	**3 **^**′ **^**Near Seq 30 bp**	**Codon position**	**Protein residue**	**Amino acid position**
**rs1063114**	Exon 8	agactgtgatgtcataattaatgaattgtg	**A/T**	cataggttaggtggtgaatatgccaaactt	**3**	Ter/Cys [*/C]	**490**
[C_9638456_10]			ancestral allele: **T**				
**rs1063111**	Exon 8	ttgatgtagagcttcttggagactgtgatg	**A/T**	cataattaatgaattgtgtcataggttagg	**2**	**Asp/Val [D/V]**	**484**
[C_9638445_10]			ancestral allele: **T**				
**rs1063112**	Exon 8	atgtagagcttcttggagactgtgatgtca	**C/T**	aattaatgaattgtgtcataggttaggtgg	**2**	**Thr/Ile**	**485**
[SIRT1-A485]			ancestral allele: **T**			**[T/I]**	
**rs35224060**	Exon 9	ggagatgatcaagaggcaattaatgaagct	**A/G**	tatctgtgaaacaggaagtaacagacatga	**1**	**Ile/Val**	**731**
[C_25611590_10]			ancestral allele: **n.a.**			**[I/V]**	
**rs3740051**	promoter	agccgcctccttttgcctctcttcctactt	**A/G**	ttaacaaaacagaacgactatccaacgtat	**-**	**-**	**-**
[C_27471644_10]							
			ancestral allele: **A**				
**rs2236319**	Intron 4	agggatgtcagtctgatggagaaattgggt	**A/G**	tttgttagatctttatgagaaactggaaac	**-**	**-**	**-**
[C_15954063_10]			ancestral allele: **A**				

bp: base pair; dbSNP: Database of Single Nucleotide Polymorphisms.

## Competing interests

The authors declare that they have no competing interests.

## Authors’ contributions

SVM conducted the study, designed and carried out the experiments, wrote the manuscript. BR carried out the experiments. CS carried out the experiments. CLD was responsible for the experimental design and statistical analysis. SL was responsible for the experimental design. UM was responsible for the study design, statistical analysis and writing of the manuscript. All authors read and approved the final manuscript.

## References

[B1] PalmerKTCoggonDBendallHEPannettBGriffinMJHawardBMHand-transmitted vibration: occupational exposures and their health effects in Great Britain1999Suffolk: HSE Books, Sudbury

[B2] BologniaJLJorizzoJLRapiniRPDermatology: 2-Volume Set2007St. Louis, MO: Mosby

[B3] TaylorWThe vibration syndrome1974London: Academic

[B4] DupuisHWirkung mechanischer Schwingungen auf das Hand-Arm-System1982BAU Dortmund: Literaturanalyse

[B5] DupuisHRiedelSKonietzko J, Dupuis HHandbuch der ArbeitsmedizinVibrationsbedingtes Vasospastisches Syndrom VS (BK 2104)1999Landsberg: Ergomed Verlag342

[B6] DongCYoonWGoldschmidt-ClermontPDNA methylation and atherosclerosisJ Nutr20021322406S2409S1216370110.1093/jn/132.8.2406S

[B7] LundGAnderssonLLauriaMLindholmMFragaMFVillar-GareaABallestarEEstellerMZainaSDNA methylation polymorphisms precede any histological sign of atherosclerosis in mice lacking apolipoprotein EJ Biol Chem2004279291472915410.1074/jbc.M40361820015131116

[B8] KimMKwonHLeeYBaekJHJangJELeeSWMoonEJKimHSLeeSKChungHYKimCWKimKWHistone deacetylases induce angiogenesis by negative regulation of tumor suppressor genesNat Med2001743744310.1038/8650711283670

[B9] EdelsteinLPanACollinsTChromatin modification and the endothelial-specific activation of the E-selectin geneJ Biol Chem2005280111921120210.1074/jbc.M41299720015671023PMC1382061

[B10] FishJMatoukCRachlisALinSTaiSCD’AbreoCMarsdenPAThe expression of endothelial nitric-oxide synthase is controlled by a cell-specific histone codeJ Biol Chem200228024824248381587007010.1074/jbc.M502115200

[B11] WuJIwataFGrassJOsborneCSElnitskiLFraserPOhnedaOYamamotoMBresnickEHMolecular determinants of NOTCH4 transcription in vascular endotheliumMol Cell Biol2005251458147410.1128/MCB.25.4.1458-1474.200515684396PMC548019

[B12] CollinsFSBrooksLDChakravartiAA DNA polymorphism discovery resource for research on human genetic variationGenome Res1998812291231987297810.1101/gr.8.12.1229

[B13] BarnesMRSNP and mutation data on the web - hidden treasures for uncoveringComp Funct Genomics20023677410.1002/cfg.13118628874PMC2447234

[B14] ZschoernigBMahlknechtUSIRTUIN 1: regulating the regulatorBiochem Biophys Res Commun200837625125510.1016/j.bbrc.2008.08.13718774777

[B15] ZschoernigBMahlknechtUCarboxy-terminal phosphorylation of SIRT1 by protein kinase CK2Biochem Biophys Res Commun200938137237710.1016/j.bbrc.2009.02.08519236849

[B16] MahlknechtUVoelter-MahlknechtSChromosomal characterization and localization of the NAD + −dependent histone deacetylase gene sirtuin 1 in the mouseInt J Mol Med20092324525219148549

[B17] Voelter-MahlknechtSMahlknechtUCloning, chromosomal characterization and mapping of the NAD-dependent histone deacetylases gene sirtuin 1Int J Mol Med200617596716328012

[B18] BlanderGGuarenteLThe Sir2 family of protein deacetylasesAnnu Rev Biochem20047341743510.1146/annurev.biochem.73.011303.07365115189148

[B19] VaqueroAScherMLeeDErdjument-BromageHTempstPReinbergDHuman SirT1 interacts with histone H1 and promotes formation of facultative heterochromatinMol Cell2004169310510.1016/j.molcel.2004.08.03115469825

[B20] TaiSRobbGMarsdenPEndothelial nitric oxide synthase: a new paradigm for gene regulation in the injured blood vesselArterioscler Thromb Vasc Biol20042440541210.1161/01.ATV.0000109171.50229.3314656742

[B21] MattagajasinghIKimCSNaqviAYamamoriTHoffmanTAJungSBDeRiccoJKasunoKIraniKSIRT1 promotes endothelium-dependent vascular relaxation by activating endothelial nitric oxide synthaseProc Natl Acad Sci U S A2007104148551486010.1073/pnas.070432910417785417PMC1976244

[B22] EngelNMahlknechtUAging and anti-aging: unexpected side effects of everyday medication through sirtuin1 modulationInt J Mol Med20082122323218204789

[B23] SmigielskiEMSirotkinKWardMSherrySTdbSNP: a database of single nucleotide polymorphismsNucleic Acids Res20002835235510.1093/nar/28.1.35210592272PMC102496

[B24] International HapMap ConsortiumThe International HapMap ProjectNature200342678979610.1038/nature0216814685227

[B25] De La VegaFMDaileyDZiegleJWilliamsJMaddenDGilbertDANew generation pharmacogenomic tools: a SNP linkage disequilibrium Map, validated SNP assay resource, and high-throughput instrumentation system for large-scale genetic studiesBiotechniques20025248505412083398

